# The Role of Knowledge Creation-Oriented Convolutional Neural Network in Learning Interaction

**DOI:** 10.1155/2022/6493311

**Published:** 2022-03-16

**Authors:** Hongyan Zhang, Xiaoguang Luo

**Affiliations:** ^1^School of Economics and Management, Harbin University of Science and Technology, Harbin, Heilongjiang, China; ^2^Department of Management, Harbin Finance University, Harbin, Heilongjiang, China; ^3^School of Economics and Management, Harbin University of Science and Technology, Harbin, Heilongjiang, China

## Abstract

When convolutional neural network (CNN) applications have different tasks in the source domain and target domain, but both have labels, it is easy to ignore the difference between the source domain and target domain by using the current traditional method, and the recognition effect of image features is not ideal. This paper proposes a deep migration learning method based on improved ResNet based on existing research to avoid this problem. This method extracts high-order statistical features of images by increasing the number of network layers for classification when performing model transfer learning. The ImageNet dataset is used as the source domain, and a Deep Residual Network (DRN) is used for model transfer based on homogeneous data. Firstly, the ResNet model is pretrained. Then, the last fully connected layer of the source model is modified, and the final deep model is constructed by fine-tuning the network by adding an adjustment module. The impact of content differences between datasets on recognizing transfer learning features is reduced through model transfer and deep feature extraction. The deep transfer learning methods after improving ResNet are compared through experiments. The identification algorithm is based on Support Vector Machine (SVM), the deep transfer learning method on Visual Geometry Group (VGG)-19, and the deep transfer learning method based on Inception-V3. Four experiments are performed on MNIST and CIFAR-10 datasets. By analyzing the experimental data, ResNet's improved deep transfer learning method achieves 97.98% and 90.45% accuracy on the MNIST and CIFAR-10 datasets, and 95.33% and 85.07% on the test set. The accuracy and recognition accuracy on the training and test sets have been improved to a certain extent. The combination of CNN and transfer learning can effectively alleviate the difficulty of obtaining labeled data. Therefore, the application of a CNN in transfer learning is significant.

## 1. Introduction

Although computer learning algorithm has many advantages and is more and more widely used in various fields, it requires high data collected. When the computer is running, it must meet a condition that the training set and the test set must be independent of each other but their distribution must be the same [1]. Once the data collected do not meet the above requirements, it is necessary to recollect the data and determine whether the data collected meet the requirements. This process will undoubtedly waste a lot of manpower and material resources. Therefore, people hope to avoid this problem in practical application. In the field of computer learning, transfer learning mainly uses the difference between source domain and target domain to calibrate the data. Therefore, it does not need to spend a lot of time on data collection, which also avoids the shortcomings of computer learning algorithms [2].

Transfer learning has received attention since 1995, and its goal is to use knowledge learned from one environment to help learning tasks in a new environment. The transfer learning of Deep Convolutional Neural Networks (DCNN) studies how to complete the transfer learning task of source domain and target domain through DCNN. Due to the popularity of DCNN in various fields, many transfer learning methods for DCNN have been proposed one after another. According to the techniques used in transfer learning, these methods are divided into four categories: instance-based DCNN transfer learning, mapping-based transfer learning for DCNN, model-based transfer learning for DCNN, and adversarial-based transfer learning for DCNN [3, 4]. Instance-based DCNN transfer learning generally sets different weights for different samples through a particular weight allocation strategy and then cooperates with DCNN for training. Mapping-based transfer learning for DCNN refers to mapping data from source and target domains to a new feature space in which data from both disciplines are equally distributed. At present, many network models have been pretrained in the source domain, and their network structure and weight parameters are known. The network-based DCNN transfer learning method transfers part of the model structure and parameters to the target domain for retraining or prediction. Adversarial-based DCNN transfer learning utilizes the adversarial technique of generative adversarial networks to find transferable features suitable for the target domain by aligning the source and target domains [5].

According to related research, whether the source and target domains have labels and whether the tasks of the source and target domains are the same, these conditions affect the techniques used in transfer learning. Moreover, the transfer learning methods under different conditions are very other. Therefore, this study proposes a transfer learning method using DCNN under different conditions for whether the source domain and target domain labels are the same or not. Both the source domain and the target domain have labels but distinct tasks. A deep transfer learning method based on improved ResNet is proposed to enhance the feature recognition ability of deep model transfer learning, which enhances the feature recognition ability of the model by increasing the number of network layers. The algorithm effectively combines and transforms the model construction and training methods based on transfer learning, avoids the problem of reduced target domain feature recognition due to differences in the content of the data sets, and improves the recognition rate.

## 2. Materials and Methods

In recent years, DCNN has become a hot topic in pattern recognition and has broad application prospects. DCNN is an end-to-end strategy, and its powerful learning ability is due to the use of multiple feature extraction stages, which can automatically learn representations from data. However, training a DCNN requires many training samples and the training set and test set to satisfy the same data distribution and in many practical application recognition tasks. It is not easy to obtain many training samples, such as the smoke data set. Currently, smoke data is only available in trace amounts with labels. Therefore, the problem of deep feature extraction for small samples has become a hot research topic. The focus is on performing task recognition with a DCNN under a small training sample.

Transfer learning aims to use the model trained in the source domain to transfer to the target domain for education, avoiding the same distribution condition commonly required in traditional machine learning. The distribution difference between the source and the target domain can be reduced for knowledge transfer through transfer, thereby realizing data calibration. The combination of transfer learning and DCNN can effectively solve the problem of insufficient sample data and avoid the difficulty of developing deep models. However, due to the different tasks in the source and target domains, the transfer learning method will reduce the feature recognition ability due to the content difference between the two datasets, resulting in a decrease in the recognition rate.

Given the low similarity between the source and target domains, this chapter uses the DRN, combined with transfer learning. It proposes a transfer learning method based on improved ResNet. During model migration, the feature recognition ability of the model is enhanced by increasing the number of network layers. Firstly, ResNet is transferred to the target dataset, and only the classifier layer is trained, resulting in an intermediate model. Secondly, the medium model is improved, and an adjustment module is added based on the intermediate model. The target data set is trained, and only the adjustment module needs to be prepared. Then, the transfer learning model based on the improved ResNet is constructed. The experiments use standard datasets, and the recognition accuracy can be improved by creating a deep transfer learning network.

### 2.1. Related Concepts and Analysis

### 2.2. Knowledge Creation Theory

With the development of contemporary scientific and technological revolution, knowledge creation ability has become one of the decisive factors of competition among countries [6]. Although the current attention to knowledge creation is increasing, its definition is still vague. From the relatively simple literal meaning, knowledge creation refers to the creation of a new theory or law through certain reasoning analysis or experimental research [7]. However, in the field of constructive learning, the definition of knowledge creation is slightly different from the above definition. Relevant researchers believe that the process of knowledge construction is actually the knowledge creation. The knowledge creation mentioned here does not require students to put forward the “Law of Universal Gravitation” like Newton, or to create nine world-famous symphonies like Beethoven, but requires students to put forward new ideas according to their existing knowledge [8]. Therefore, the knowledge creation ability mentioned refers to the process that students can migrate through the existing knowledge system, discover new problems, and constantly think and innovate [9].

According to relevant international regulations, knowledge is divided into 6 categories, as shown in Figure 1.

#### 2.2.1. CNN

The composition of CNN is shown in Figure 2.

Convolution operation is to identify the features of the input data by convolution kernel [10]. The convolution kernel and the grid structure of the input data are relatively regular and can be stored in the form of multidimensional arrays. The size of convolution kernel is theoretically arbitrary, but it is often smaller than the input data [11].

Convolution operations are effective for certain types of data. They use the invariant data attributes such as spatial local characteristics and translation invariance to analyze the input data. Convolution operation uses the above two data attributes to identify the characteristics of the input data through convolution kernel [12]. In addition, since the convolution kernel used in the process of input data is the same, compared with the traditional neural network, CNN involves fewer parameters in the analysis of data, making the analysis process simpler. The above concept is called parameter sharing [13]. The traditional full connection layer will involve a large number of parameters, so the use of relatively small convolution kernel can reduce the number of parameters. The above concept is called sparse connection [14].  Figure 3 presents the basic structure of CNN.

In CNN, convolution operation is usually nonlinear operation and pooling operation, which is an effective framework for identifying data features. Nonlinear operation ensures that the properties of the neural network are nonlinear by nonlinear operation of the input data. Pooling operation reduces the output of data by further simplifying the input data. However, those pooling operations still highlight key features of data. For example, if a user wants to retain key features in a local area, the data can be processed using maximum pooling operations. The operation of the convolution operator at the initial development on the real value can be theoretically expressed by

(1) $$\begin{array}{c} y\left(\left(z\right)\right)=\left(x*w\right)\left(z\right)=\int x\left(t\right)w\left(z-t\right)\text{d}t. \end{array}$$

In (1), *x*(*t*) is input values on the *t* position and *w* is convolution kernel. Equation (1) can be regarded as the weighted average of *w* in the whole neighborhood of *x*. If the input data are multidimensional (e.g., image signal), the above function can be replaced by multivariate. If the input data are discrete, the above operation can be replaced by summation. For example, the convolution operation using two-dimensional kernel *w* on two-dimensional image *x* can be expressed by

(2) $$\begin{array}{c} y\left(m,n\right)=\left(x*w\right)\left(m,n\right)=\sum_{i,j}x\left(i,j\right)w\left(m-i,n-j\right). \end{array}$$

Equation (2) shows that the center of the convolution kernel is placed on the corresponding pixel position for the pixel value of the coordinate (*m*, *j*), and the sum of the corresponding pixel product and the overlapping parameters is calculated. Finally, the output on the position (*m*, *n*) is obtained. This process is the basis of convolution stage operation in CNN. Through this operation, different features of the input data can be extracted.

#### 2.2.2. DCNN

In recent years, with the wide application of CNNs, more and more researchers have begun to focus on the CNNs with better design performance. Meanwhile, the topological structure processed by CNN is also more complex, which lays the foundation for the establishment of DCNN [5]. The biggest difference between DCNN and previous neural networks is its convolution layer [15].  Figure 4 presents the structure diagram of DCNN.

According to the different direction of data propagation, DCNN training can be divided into two processes: forward and backward. When data propagates forward, it needs to calculate the data values needed to activate each layer of the network and then propagates backwards from the input layer until it reaches the final output layer. On the contrary, when the data propagate backward, it propagates layer by layer from the last layer forward according to the calculated gradient. When this process is finished, it will calculate the gradient of each layer, and meantime, it needs to update the network parameters, and through the calculation of the partial derivative of the loss function for the network parameters, the network parameters are constantly updated. The specific calculation process is as follows: if there is a training set *X*={(*x*^(1)^, *y*^(1)^),…, (*x*^(*m*)^, *y*^(*m*)^)}, where the number of samples is *m*, a single sample is *x*^(*l*)^, and the labels corresponding to each sample represented by *y*^(*l*)^, then the loss function of the sample can be calculated by

(3) $$\begin{array}{c} J\left(W,b;x,y\right)=\frac{1}{2}{\left\|h_{W,b}\left(x\right)-y\right\|}^{2}. \end{array}$$

The loss function for the entire dataset can be calculated by

(4) $$\begin{array}{c} J\left(w,b\right)=\frac{1}{m}\sum_{i=1}^{m}\left({\left\|h_{w,b}\left(x^{\left(i\right)}\right)-\left(y^{\left(i\right)}\right)\right\|}^{2}\right)+\frac{\lambda }{2}\sum_{l=1}^{n_{l}-1}\sum_{i=1}^{s_{l}}\sum_{j=1}^{s_{l}+1}{\left(w_{ji}^{\left(l\right)}\right)}^{2}. \end{array}$$

In equation (4), the error generated by all samples in the sample set is calculated. The second function after the equation is to control the weight range in the process of network training. The trade-off between mean square error and regularization term can be controlled by parameter.

After the loss function of the entire dataset is calculated through (4), the gradient needs to be calculated and the network parameters need to be updated. When updating the weights *W* and offset *b*, the gradient descent method is used. The specific calculation equation is as follows:

(5) $$\begin{array}{c} W_{ij}^{\left(l\right)}=W_{ij}^{\left(l\right)}-\alpha \frac{\partial }{\partial W_{ij}^{\left(l\right)}}J\left(W,b\right),\\ b_{i}^{\left(l\right)}=b_{i}^{\left(l\right)}-\alpha \frac{\partial }{\partial b_{i}^{\left(l\right)}}J\left(W,b\right). \end{array}$$

#### 2.2.3. DCNN

DCNN has seen various improvements since the success of AlexNet in 2012. Since the number of layers of DCNN is often significant, it brings a large number of parameters that need to be learned. If it is not handled correctly, it will bring about overfitting problems. It is generally controlled effectively from the data itself and the optimization of model training to prevent the overfitting of the model. The following methods are often used as techniques to improve DCNN.

1. Data Enhancement. The successful application of DCNN relies on the massive availability of labeled data. However, there is often insufficient data, so how to obtain more data is the key to the problem. If it is used to collect or label information manually, it will cost a lot. Data augmentation is used to solve such problems. Data augmentation refers to using existing data to obtain more data without substantially increasing the data. The existing datasets are used as common geometric transformations to get more data, such as rotation, sampling, and movement.
2. Weight Initialization. Meticulous weight initialization is the mainstream of current DCNN training techniques. When the network is deep, the neural network is susceptible to the initial weight, and its distribution directly affects the motor nerve of the network. Therefore, the initial weight distribution needs to be adjusted to avoid vanishing and exploding gradients. Bias will generally be initialized to zero.
3. Batch Standardization. Data preprocessing is an essential model training process, which needs to adjust the data to a standard normal distribution. However, in training a DCNN, the data needs to pass through a multilayer network, and the weights and biases can affect the accuracy of the final output. A batch normalization (BN) method is proposed to deal with internal covariance shifts in feature maps to alleviate the above phenomenon. Internal covariance shifts are changes in the distribution of remote unit values that force the learning rate to a minimum, slowing down the convergence of the model training process and requiring careful initialization of parameters.

### 2.3. Model Construction

In traditional CNN, as the depth of the network continues to increase, gradient vanishing and gradient explosion are unavoidable. In this case, since the recognition rate gradually reaches saturation, continuing to increase the depth of the network will cause the recognition rate to drop, which is caused by the gradient degradation problem generated during the training process. Therefore, scholars have proposed the DRN, an extremely DCNN model. On the one hand, it avoids the difficulties of gradient disappearance and gradient explosion, and on the other hand, it better solves the problem of gradient degradation. The building blocks of ResNet are shown in Figure 5.

Let *F*(*x*) be the mapping defined by the two convolutional layers, and the output function becomes *F*(*x*)+*x* after adding shortcut connections. Assuming that *H*(*x*) represents the ideal output of the network after the input sample *x*, in the traditional CNN (Convolution Neural Networks), there is *H*(*x*)=*F*(*x*). This traditional representation does not preserve the information of the original *x*. In the residual learning structure, there is *H*(*x*)=*F*(*x*)+*x*, and *F*(*x*) is called the residual function. Here, the residual network no longer adjusts the weights to fit the function *H*(*x*), but instead fits the residual function *F*(*x*). In theory, if *H*(*x*) can be approximated by *F*(*x*), then it can also be approximated by *F*(*x*)+*x*. When the DRN automatically extracts features, it only needs to set *F*(*x*)=0 to complete an identity mapping *H*(*x*)=*x*. The network is used to fit a certain function *F*(*x*)=0, which is easier than fitting a *H*(*x*) function. When fitting *F*(*x*)=0, both weights and biases approach 0.

Unlike other DCNN, ResNet utilizes shortcut connections to achieve data superposition between input and output. Under the shortcut connection, the number of parameters and computational complexity of the network does not increase, so the number of layers of ResNet can maintain a fast calculation speed even in a serious case. ResNet solves the problem of gradient degradation by increasing the connection across layers. ResNet optimization relative to other DCNNs also uses BN between the convolution and activation functions. BN can speed up network training and prevent the gradient explosion of the network.

At present, DCNN has a thorny problem; that is, it has its corresponding labels in both source domain and target domain, but its tasks are different. The traditional method is to initialize the network parameters and then transfer learning through fine tuning. But this method does not pay attention to the fact that the content between the source domain and the target domain is not exactly the same. Therefore, in order to make up for the shortcomings of traditional methods, this paper improves ResNet and proposes a new deep transfer learning method [16, 17]. After improving ResNet, a deep transfer learning model is reframed, as shown in Figure 6.

In Figure 6, the top graph is the pretraining ResNet-34 model. The intermediate model is obtained by replacing the classifier layer. It is obtained by retaining all parameters in the convolution layer of the topmost model and replacing only the full connection layer. The following is the final model.

#### 2.3.1. Pretraining ResNet-34 Model

In migration learning, the DCNN model needs to be trained on large data sets. According to the different directions of data propagation, this training process is divided into forward propagation and backward propagation [18]. Assuming that there are *m* class *c* samples in the model training set, the single training sample is represented by (*x*^(*i*)^, *y*^(*i*)^). The forward propagation process of layer *l* can be represented by

(6) $$\begin{array}{c} x^{l}=f\left(u^{l}\right),u^{l}=w^{l}x^{i-1}+b^{l}. \end{array}$$

In (6), *x*^(*i*)^ is *n*-dimensional input sample. *y*^(*i*)^ is the sample belonging to category. *l* is network layer. *x*^(*i*−1)^, *x*^(*l*)^ are *l* layer input, output. w^l^ is convolution kernel weight. *b*^l^ is partial value. *f*(·)is activation function.

For a dataset {(*x*^(*l*)^, *y*^(*l*)^),…, (*x*^(*m*)^, *y*^(*m*)^)} with *m* samples, the loss function can be expressed by

(7) $$\begin{array}{c} J\left(w,b\right)=\frac{1}{m}\sum_{i=1}^{m}\left(\frac{1}{2}{\left\|h_{w,b}\left(x^{\left(i\right)}\right)-\left(y^{\left(i\right)}\right)\right\|}^{2}\right)+\frac{\lambda }{2}\sum_{l=1}^{n_{l}-1}\sum_{i=1}^{s_{l}}\sum_{j=1}^{s_{l}+1}{\left(w_{ji}^{\left(l\right)}\right)}^{2}. \end{array}$$

In (7), *λ* is weight attenuation coefficient. *n*_*l*_ is convolution neural network layers. *s*_*l*_ is the number of network neurons in layer *l*.

When the parameters are fine-tuned, the gradient descent method is used to minimize the overall loss function. Update each layer parameter *w*_*ij*_^(*l*)^ and *b*_*i*_^(*l*)^ through (8) and (9):

(8) $$\begin{array}{c} W_{ij}^{\left(l\right)}=W_{ij}^{\left(l\right)}-\alpha \frac{\partial }{\partial W_{ij}^{\left(l\right)}}J\left(W,b\right), \end{array}$$

(9) $$\begin{array}{c} b_{i}^{\left(l\right)}=b_{i}^{\left(l\right)}-\alpha \frac{\partial }{\partial b_{i}^{\left(l\right)}}J\left(W,b\right). \end{array}$$

In (8) and (9), *α* is learning rate. When calculating the partial derivative of the cost function, it needs to calculate the error unit of each network layer in advance. Whether DCNN model pretraining is completed can be seen by error size.

#### 2.3.2. Classifier Retraining [19]

In the process of transfer learning, the typical process based on model is from source model to intermediate model. When constructing DCNN model, it combines layer freezing method with pretraining model. The main processes are as follows.

By pretraining the parameters of Res Net model, it is necessary to use the parameters retained in the previous process to extract the data features in the next stage, which is called the initialization stage. All parameters and weight data outside the fully connected classification layer are loaded. Assuming that the target data set involved is a total of *k* classes, the last layer of the fully connected layer can be changed by the *k*-element softmax classifier. This process only trains the new classifier layer. The convolution and pooling layers in the pretraining model are frozen, which is the first stage. The whole process migrates the reserved parameters and docks the *k*-element softmax classifier in the previous stage to get the intermediate model.

#### 2.3.3. Adjust Module Retraining

Transfer learning usually freezes the weights of the top *k* layers in a pretrained model. Then, data from the target domain is used to retrain the subsequent *n* − *k* layers, a process called fine-tuning. The purpose of fine-tuning is to extract high-level features of the target domain, reduce the content difference between the source domain and the target domain, and improve the model recognition rate. Increasing the number of network layers can extract more high-level features. Therefore, the number of network layers should be appropriately increased while performing transfer learning—that is, an adjustment module should be added. In this way, the model captures specific high-order statistical features of the target domain [20].

Let *H*_*T*_(*x*) and *H*_*S*_(*x*) be the network models of the source and target domains, respectively. If the last *k* layers are only retrained, then *H*_*T*_(*x*)=*H*_*S*_(*x*) directly transfers the model trained in the source domain to the target domain for training and prediction. Although this method is feasible, it considers the differences between the source domain and the target domain. The features they extract are not exactly the same. Therefore, the features extracted from the source domain are used to identify the task of the target domain, which will reduce the feature recognition ability. The content difference between the source domain and the target domain is reduced by adding network layers. On this basis, the proposed method fully considers the characteristics of the target domain. Compared with the traditional network structure, the novelty of the proposed method is to adapt the classification task of the target domain by adding an adjustment module Δ*H*(*x*) on the source model. Such improvements extend the learning capabilities of the network. Meanwhile, the increase of network depth helps extract deeper features, thereby improving the classification accuracy of the target domain. The relationship between *H*_*T*_(*x*) and *H*_*S*_(*x*) is shown in

(10) $$\begin{array}{c} H_{T}\left(x\right)=H_{S}\left(x\right)+\Delta H\left(x\right). \end{array}$$

The first few layers of DCNN contain more general characteristics, such as edge information and color information. This is very useful for many tasks. However, the feature learning of the last layers of DCNN focuses on high-level features. The purpose of increasing the number of network layers is to extract high-level semantic features of the target domain. Therefore, the number of network layers is usually chosen to grow at the end of the model.

In Figure 6, the last two layers of the intermediate model are the mean pooling layer and the softmax classifier layer, respectively. In training the final model, it is only necessary to adjust the module Δ*H*(*x*) for backpropagation, and the rest of the network layer parameters are frozen. Therefore, the input and output dimensions of the module must be the same to keep the network model reasonable. A major feature of the residual structure is that the input and output dimensions remain the same after the 3^∗^3 convolution kernel. The biggest difference from other DCNNs is that ResNet uses shortcut connections to achieve data superposition between input and output. In this connection mode, the network's parameter amount and computational complexity are not increased due to the increase of network layers. Therefore, the structure of ResNet can maintain a fast computation speed even in the deep case. To sum up, the residual block is selected as the adjustment module.

The adjustment module (residual block) employs two consecutive convolutional layers with a filter size of 3^∗^3. A BN layer and a ReLu activation function layer are added after each convolutional layer so that the image undergoes two nonlinear activation function calculations. Let loss be the loss value obtained by the cost function, and the cost function is *l*(·). loss is shown in

(11) $$\begin{array}{c} \text{loss}=l\left(o_{n}\right). \end{array}$$

*o*_*n*_ is the output feature map of the *n*th layer of the network. *i*_*n*_ is the input of the *n*th layer and the output of the *n* − 1th layer. *w*_*n*_ and *b*_*n*_ are the connection weights and bias terms of the *n*th layer, respectively. The output feature map of each layer is shown in

(12) $$\begin{array}{c} o_{n}=f_{n}\left(i_{n},w_{n},b_{n}\right). \end{array}$$

The shortcut connection directly spans two convolutional layers, converting the input to the output through an identity map. The calculation of the gradient of each layer is

(13) $$\begin{array}{c} \frac{\partial o_{n}}{\partial i_{n}}=\frac{\partial \left(i_{n}+f_{n}\left(i_{n},w_{n},b_{n}\right)\right)}{\partial i_{n}}=1+\frac{\partial f_{n}\left(i_{n},w_{n},b_{n}\right)}{\partial i_{n}}. \end{array}$$

In the ResNet-34 model, the input image size is 224×224. The output after the last residual block is *Y*_33_. After being added to the adjustment module (two convolutional layers), *Y*_34_=*σ*(*W*_34_*Y*_33_+*b*_34_) and *Y*_35_=*σ*(*W*_35_*Y*_34_+*b*_35_) are output separately, where *σ* is the ReLu activation function and *W*_34_, *b*_34_, *W*_35_, *b*_35_ are the parameters that need to be trained in the target domain.

### 2.4. Model Analysis

The time complexity of CNN training can be expressed by

(14) $$\begin{array}{c} \text{Time}∼O\left(\sum_{l=1}^{D}M_{l}^{2}\cdot K_{l}^{2}\cdot C_{l-1}\cdot C_{l}\right). \end{array}$$

In (14), *D* is convolution neural network depth. *l* is the *l*th convolution layer of CNN. *M*_*l*_ is the edge length of the feature map obtained by each convolution kernel in the *l*th convolution layer. *K*_*l*_ is the edge length of each convolution kernel in the *l*th convolution layer. *C*_*l*_ is the number of output channels contained in the *l*th convolution layer. *C*_out_ is the number of convolution kernels contained in the *l*th convolution layer.

(14) indicates that *M*^2^, *K*^2^, *C*_in_, and *C*_out_ directly determine the time complexity of a CNN for training. The spatial complexity of training a CNN can be expressed by

(15) $$\begin{array}{c} \text{Space}∼O\left(\sum_{D}^{l=1}K_{l}^{2}\cdot C_{l-1}\cdot C_{l}\right). \end{array}$$

*K* ^2^, *C*_in_, and *C*_out_ determine the spatial complexity.

### 2.5. Experimental Setup

The method studied is applied to the identification task to analyze the advantages of this algorithm in the application of migration learning. Four comparative experiments are set up in this experiment, namely, the recognition algorithm based on Support Vector Machine (SVM), the deep migration method based on VGG-19, Inception-V3, and ResNet-34, respectively. These are called SVM, VGG19-migration, Inception-V3-migration, and Res Net34-migration, respectively.

The experimental environment used is Windows 10 Professional edition with memory of 4 GB and processor of 2.5 GHz Intel i5 CPU. The experiment is carried out in the model with Tensor Flow framework. The task recognition experiments are carried out on two large datasets, MNIST and CIFAR-10, respectively.

MNIST dataset is a digital database established by New York University. This database contains 10 categories, of which the test set and the training set contain 10,000 and 60,000 pictures of 28^∗^28. The CIFAR-10 dataset contains 60,000 color images with a size of 32^∗^32 and 6,000 images in each category. Among them, the test dataset and the training dataset contain 10,000 and 60,000 images, respectively. The source domain of this experiment uses Image Net large dataset [21]. Image Net dataset contains a large number of image data, which currently ranks first in the world. It is established by Fei-Fei Li et al., and the image category is as high as more than 1000, which provides a strong guarantee for the construction of CNN-based migration learning model.

Batch Gradient Descent (BGD) is used as the optimization algorithm when training the model, where the number of training samples per batch is set to 64 [22]. The total number of iterations is 26 epochs, and the training samples are randomly scrambled again after one generation is completed. The learning rate is set using a step-down strategy, and its initial value is set to *e*^−4^ according to the empirical value. It decreases once every 10 epochs with a decreasing factor of 0.1 [23]. The training parameters of the CNN are shown in Figure 7.

In this experiment, the following three criteria are used to evaluate the effect of the experimental method: Training Accuracy, Test Accuracy, and Loss Function [24–26]. The definition of training set accuracy is as follows:

(16) $$\begin{array}{c} \text{TrainAcc}=\frac{\text{TrainImagesCurrently}}{\text{TrainImages}}. \end{array}$$

In (16), TrainImagesCurrentlyis the number of correct images recognized in the training set; TrainImagesis the total number of images in training set. The accuracy of test set can be defined by

(17) $$\begin{array}{c} \text{TestAcc}=\frac{\text{TestImagescurrently}}{\text{TestImages}}. \end{array}$$

In (17), TrainImagesCurrentlyis the number of correct images recognized in the test set; TrainImagesis the total number of images in the test set. The value of test accuracy can represent the recognition effect.

When using the equation to represent the loss function, cross-entropy loss function is used. In the training process, the error caused by cross-entropy is minimized as follows:

(18) $$\begin{array}{c} L=-\sum_{k=1}^{n}\overset{c}{\underset{i=1}{\sum }}t_{ki}\log\left(y_{ki}\right). \end{array}$$

In (18), *t*_*ki*_is the probability of *k* samples in category *i*. *y*_*ki*_is the probability of class *i* after the prediction of sample *k* using the model.

## 3. Results

It is applied to the recognition task to verify the transfer performance of the proposed algorithm. This chapter has four comparative experiments: the recognition algorithm of Support Vector Machine (SVM), the deep transfer learning method based on VGG-19, the deep transfer method based on Inception-V3, and the deep transfer method based on ResNet-34. For the convenience of description, they are called SVM, VGG19-transfer, Inception-V3-transfer, and ResNet34-transfer in sequence. Algorithms based on transfer learning all use the method of replacing the classification layer and retraining the last two layers while retaining part of the feature extraction ability of the source model.

### 3.1. Comparison of Effect between Different Algorithms

Based on the model training parameters listed in Figure 5 and the data set divided in the previous section, the experimental results obtained are shown in Table 1 and Table 2.

In Tables 1 and 2, in the classification task of small datasets, the transfer learning method based on DCNN has improved the accuracy of training and test sets compared with traditional methods. This is mainly because the automatic feature extraction method of DCNN is superior to the conventional manual feature extraction method. Comparing the three transfer learning methods based on the DCNN model, the transfer learning method based on the ResNet model has the highest recognition accuracy. The proposed method is compared with existing methods, and a tuning module is added to the model to extract high-order statistical features specific to the target dataset. Meanwhile, the adjustment module can also deepen the base-based model structure and improve the representation ability of the base network. Thus, the recognition accuracy is further enhanced. The proposed method does not suffer from training due to the deepening of the number of layers. Compared with the transfer learning method based on ResNet-34, the recognition rate is improved on both datasets. Although the number of parameters has increased by one-sixth, the training time remains the same. Compared with the transfer learning method based on VGG-19, the number of network layers is two times that of VGG-19. However, due to the advantages of the ResNet residual block, the memory consumption for training does not double, and the drop in training speed is within an acceptable range. Compared with the other four comparison methods, transfer learning increases the number of network layers. It adds the unique high-order statistical features of the target domain to reduce the impact of content differences between datasets on the feature recognition of the target domain. It is applied to two different datasets, and it has an absolute advantage in training set and test set accuracy. The test set accuracy reaches 95.33% and 85.07%, respectively.

### 3.2. Validation Accuracy and Loss Comparison of Different Algorithms

On the MNIST test set, the accuracy and loss curves of the proposed algorithm are compared with those of the traditional algorithm with the number of iterations. The drawn curves are shown in Figures 8 and 9.

On the CIFAR-10 test set, the accuracy and loss of the proposed algorithm and the traditional algorithm are compared with the variation curve of the number of iterations (epoch). The curves are shown in Figures 10 and 11.

In Figures 8–11, as the number of iterations increases, the model gradually converges, the loss gradually decreases and finally stabilizes. The model performs well without overfitting. However, the recognition accuracy on the MNIST dataset is significantly higher than that on the CIRAR-10 dataset. The loss function of the CIFAR-10 dataset at the beginning of the experiment is slightly higher than that of the MNIST dataset. The scale of CIFAR-10 is only a small dataset compared to ImageNet. Meanwhile, ImageNet's 1000 pictures are mainly derived from daily life, including animals, daily necessities, and vehicles, while CIFAR-10 has only four vehicles and six types of common animals. So, the similarity between the two datasets is low. The MNIST dataset is relatively simple, containing only handwritten digits, and the recognition process is relatively easy. In the MNIST dataset, the latter four methods gradually stabilize after a rapid rise in test accuracy in the first 20 iterations. VGG16-migration is stable at 83%–85%, Inception-V3-migration is stable at 87%–89%, ResNet34-migration is stable at 91%–93%, and our method is stable at 94%–96%.

In Figures 8 and 10, the performance of the SVM method on small datasets is significantly weaker than that based on deep transfer learning, mainly because the SVM method is data-dependent and requires a large amount of data to complete feature learning. DCNN can automatically extract features, and transfer learning can solve the problem of training deep models when data is insufficient. The combination of the two dramatically improves the accuracy of image recognition. Meanwhile, the model trained by the improved DRN has further improved performance compared with the original ResNet model.

## 4. Conclusion

Aiming at the knowledge creation task, this paper deeply studies how to apply CNN to transfer learning. Aiming at the situation that the source domain and the target domain have labels but different tasks, this paper proposes a deep transfer learning method based on improved ResNet. On the basis of the intermediate model, an adjustment module is added to extract the high-order statistical characteristics of the target dataset. Different from the traditional fine-tuning method, the method proposed has beneficial combination and transformation of the model construction and training method based on transfer learning. This avoids the problem of reducing the feature recognition ability of the target set caused by the difference in the content between the data sets, to improve the recognition rate. The experimental results on public datasets show that the proposed improved method has good recognition performance and strong generalization ability.

The proposed deep transfer learning method based on improved ResNet has a higher recognition rate when the number of target domain categories is small. The recognition rate is average when there are many target domain categories. Therefore, the next step will focus on the factor of the number of target domain categories in the deep transfer learning algorithm to enhance the practicability and robustness.

## Figures and Tables

**Figure 1:** 6W classification of knowledge.

**Figure 2:** Composition of CNN.

**Figure 3:** Basic structure of CNN.

**Figure 4:** Basic structure of DCNN.

**Figure 5:** Structure diagram of ResNet.

**Figure 6:** Transfer learning model training framework based on improved ResNet.

**Figure 7:** Model training parameters.

**Figure 8:** Verification accuracy on MNIST dataset.

**Figure 9:** Losses on MNIST dataset.

**Figure 10:** Verification accuracy on CIFAR-10 dataset.

**Figure 11:** Losses on the CIFAR-10 dataset.

**Table 1:** Performance comparison of different methods on the MNIST dataset.

Method	MNIST training set accuracy (%)	MNIST test set accuracy (%)	Parameters (million)	Training time (seconds/200 iterations)
SVM	78.25	74.86	8.7	8
VGG19-migration	88.62	85.59	139	40
Inception-V3-migration	93.15	89.96	23.2	65
ResNet34-migration	95.52	92.63	24.3	78
The method of this study	97.95	95.25	28.1	79

**Table 2:** Performance comparison of different methods on the CIFAR-10 dataset.

Method	CIFAR-10 training set accuracy (%)	CIFAR-10 test set accuracy (%)	Parameters/million	Training time (seconds/200 iterations)
SVM	74.24	69.35	8.7	9
VGG19-migration	83.21	78.63	139	41
Inception-V3-migration	87.73	83.24	23.2	72
ResNet34-migration	89.52	84.25	24.3	79
The method of this study	90.55	85.92	28.1	82

## Data Availability

The experimental data used to support the findings of this study are available from the corresponding author upon request.
